# Strategies for Medical Device Development: User and Stakeholder Perceptions

**DOI:** 10.1155/2023/6724656

**Published:** 2023-05-29

**Authors:** I-Ching Tsai, Ching-Da Wang, Peng-Ting Chen

**Affiliations:** ^1^Department of Biomedical Engineering, National Cheng Kung University, No. 1, University Road, Tainan City 701, Taiwan; ^2^International Institute of Medical Device Innovation, National Cheng Kung University, No. 1, University Road, Tainan City 701, Taiwan

## Abstract

Medical device development involves user safety, and it is governed by specific regulations. The failure of medical device developers to consider the influence of users, the environment, and related organizations on product development during the design and development process can result in added risks to the use of medical technologies. Although many studies have examined the medical device development process, there has been no systematic and comprehensive assessment of the key factors affecting medical device development. This research synthesized the value of medical device industry stakeholders' experiences through a literature review and interviews with industry experts. Then, it establishes an FIA-NRM model to identify the key factors affecting medical device development and suggests appropriate pathways for improvement. Results indicate that the development of medical devices should begin with stabilizing organizational characteristics, followed by strengthening technical capability and use environment, and finally, consideration should be given to the user action of medical devices. The results provide medical device developers with optimal development pathways and resource allocation recommendations to support developers in developing medical device development strategies as well as ensuring the safety and effectiveness of the products for end users.

## 1. Introduction

Medical devices have brought numerous benefits and contributions to human health; however, regulations and medical particularities increase the costs and sensitivity of medical device research, design, and clinical applications [1]. These situations pose considerable challenges to the developers, especially small-to-medium enterprises (SMEs) with limited operational resources [2, 3]. When the medical device industry fails to evaluate numerous medical device designs for the usability in the product development process, it can lead to various problems in their applicability and can give rise to risks owing to the insufficient consideration of human, environmental, and organizational factors [4, 5]. Therefore, medical device developers need to be aware of the various aspects of the development process and focus on human factors and compliance with medical device marketing regulations to reduce postmarket risks. However, an important research gap exists regarding how to invest limited resources in product development and how to formulate development strategies to achieve optimal healthcare benefits based on product efficiency, medical regulations, and user needs [6].

Many studies have examined various key factors in the medical device development process, including user operation [7], risks [8], effectiveness and regulation [9], and public stereotypes [10, 11]. Although research in medical device development continues to grow in the field of medical engineering, there is still a lack of a more systematic and comprehensive research framework based on stakeholder perspectives to evaluate the crucial elements of the medical device development process [12]. There is a need for empirical accounts of medical device development factors as perceived by stakeholders. This study analyzed the key factors in the medical device development process using stakeholder interviews and questionnaires. The results from this study can help medical device developers to prioritize and allocate resources to critical items in the medical device development process.

## 2. Literature Review

### 2.1. Medical Device Innovation Challenge

The growing demand for healthcare has made medical devices increasingly important in the healthcare industry. Countries classify medical devices according to their associated “user risk” as a basis for quality and safety management, regulatory control, or market licensing. Owing to the particularity of the medical industry and devices, governments around the world have clear classifications and strict specifications for the development and marketing of medical devices. Such regulations make the design, development, and market planning of this industry more challenging than those of general commodities [6]. One of the problems of medical device usage involves the medical device developer's failure to consider fully the application status of a product during the product design and development process, thereby resulting in equipment inapplicability. This problem may be due to a mismatch between user characteristics, product interface, and functions or the usage environment, which may affect users' cognition or cause operation errors, thereby leading to risks and injuries [13]. Overall, the ability to effectively integrate input from developers, organizations, and users in the early stages of medical device development to evaluate product design, confirm usability and save costs to develop safe and effective medical device products will provide sustainable benefits to developers and users.

### 2.2. Medical Device Development Considerations

The main purpose of a medical device is to meet indications for use and user needs. Medical device developers are often unable to understand the benefits of focusing on human engineering in the development of medical devices due to their inability to implement user involvement in the design process [14]. Therefore, developers must provide product education and training to improve operation skills and increase user confidence and trust in products [15]. In addition to incorporating human behaviour, capabilities, and limitations into the design of medical product systems, it is crucial to take into account individual user differences [16]. This includes technical knowledge, experience, and education.

Medical devices can be used in clinical or nonclinical settings, such as community homes and public settings [17]. Numerous factors related to the environment, organizational characteristics, and user status can affect the use of a medical device [18]. In the development process, the characteristics of an intended use environment (e.g., time, pressure, lighting, noise, temperature, and physical layout) can help developers understand the operation of a product and can optimize the use efficiency [19, 20] as well as improve safety and effectiveness. The development of medical devices requires consideration of the opinions of different stakeholders, the management, and the culture that can be critical to the success of the product. A variety of factors can influence the product development strategy of medical device developers, including cost control, professional manpower, budget availability, and performance expectations [21]. Given the particularity of medical devices, market strategies should consider social backgrounds, reimbursement processes, and regulatory policies [9].

This study identifies four dimensions of medical device development, including user action (UA), technical capability (TC), use environment (UE), and organizational characteristic (OC), to comprehensively assess the key factors of medical device development as a piece of advice for medical device development and medical industry.

## 3. Research Design

After conducting a literature review and examining case studies of medical device development, this study gathered specific information that influenced medical device development. For the professional experience data collection, semistructured interviews with key stakeholders were used. Key stakeholders include two managers of auditing organisations, a CEO of a consultant company, two managers of a government agency, and a product manager of a medical device company. The interview included open-ended questions, focusing on the process of medical device development and key factors. From the interviews, key aspects and factors related to medical device development were extracted and used to design questionnaires. The questionnaires were distributed among experts and their responses were recorded. The DEMATEL method was employed to analyze the questionnaire data, resulting in the establishment of a FIA-Network Relationship Map (NRM) model. The outcomes of this analysis demonstrate the importance and interaction degree for each key factor. Finally, based on the results of the FIA and NRM, suggestions were proposed for the development of the medical device development process (Figure 1).

### 3.1. Participants

The questionnaire design was based on a literature review and content analysis of expert interviews. The questionnaire investigates the background of the respondents, including their age, work experience, professional knowledge, and the organization they work for, to confirm that the respondents conform to the current study on the medical device development process. After the questionnaire was distributed, a total of 65 valid samples were collected. They work in different professions related to health care and medical equipment. Among the medical device developers that we surveyed, 23 (36.0%) were from medical profession background, 32 (49%) were engineering expertises (including technical staff and managers), and 10 (15%) were from regulatory expertises. The respondents included 48 males (74%) and 17 females (26%). The average of seniority distribution of the respondents in the biomedical industry was 9.1 years, 78% are above 5 years, and 40% are above 10 years. The study also examined the level of medical device risk involved in the development experience of the respondents, including 5 (8%) who were involved in Class I risk, 33 (50%) who were involved in Class II risk, and 27 (42%) who were involved in Class III risk.

### 3.2. Content Analysis

The content analysis uses qualitative or quantitative data and involves methods of induction or deduction. Content analysis, which is also known as text or literature analysis, converts qualitative data into quantitative data for analysis. The value of content analysis lies in its utilization of system objective and quantitative methods to classify statistics. The hidden content of records can be systematically organized and visualized based on the narrative interpretation of the numbers in the categories. Content analysis methods are applicable when sorted verbal information is critical to the research [22, 23].

Content analysis is an objective and systematic method for investigating and analyzing the content of documents and clearly describing the content of the communication. Moreover, it can analyze various languages and features in communication content [24]. The possibility of exploring a particular property of information can assist the prompt deduction of meaning. Additionally, the content analysis examines and analyzes communications to measure variables quantitatively, objectively, and systematically. Beneficial and simple, content analysis has been used in numerous aspects of scientific research for over six decades. The hypothesis of the present study states that the most frequently mentioned words reflect the biggest problem. Content analysis involves three steps, namely, unit coding, sampling, and validity analysis [25, 26].

The experts interviewed in this study were experienced in the development, management, and use of medical devices and provided valuable advice during the interviews. Content analysis was used to analyze the interviews.

### 3.3. DEMATEL Method

The DEMATEL method can be used to study and solve complex and interwoven problem sets [27]. The DEMATEL method enabled the researchers to understand specific problems and interweave clusters of problems as well as to better identify possible solutions through hierarchical structures. Recent studies have used DEMATEL techniques to solve complex problems, such as the analysis of smart product service systems [28], probabilistic safety analysis of process systems [29], pharmaceutical manufacturing [30], and hospital performance management [31]. This method differs from traditional methods in that an NRM can identify interdependence among system elements through causal graphs. In this research, the DEMATEL method was applied to constitute NRMs to investigate whether the development processes of medical device design interact with one another or they are independent. The concept of the DEMATEL method is as follows [27]. Calculate the average matrix: first, organize actors through the questionnaire and obtain interactions among the factors. Each respondent will be asked to assess the direct impact of any two factors with an integer score ranging from 0 to 4, (0 = “no influence,” 1 = “low influence,” 2 = “medium influence,” 3 = “high influence,” and 4 = “extreme strong influence”). The next step is to establish the initial influence matrix: The impact between two pairs of factors will be compared in the survey questionnaire. *X*_*ij*_ indicates the extent to which a respondent considered factor *i* affecting factor *j*, and the diagonal of the matrix shows the influence of the factor on itself, it will be set to 0 when there is no influence.

The next step is to establish the normalized direct-influence matrix: A normalized datum is the maximum of row vectors and the sum of column vectors. The normalization influence matrix is denoted by *M*, and the normalized datum is set to *s*. *M* and *s* can be calculated as follows:

(1) $$\begin{array}{c} M=sA,s\;>0\text{,} \end{array}$$

(2) $$\begin{array}{c} s=\frac{1}{\max_{ij}\left(\max_{1\leq i\leq n}\sum_{j=1}^{n}a_{ij},\max_{1\leq j\leq n}\;\sum_{i=1}^{n}a_{ij}\right)}\text{.} \end{array}$$

To calculate the indirect-influence matrix, the indirect-influence matrix is set to IM. The indirect-influence matrix can be gained by directly affecting the value of matrix (*M*) calculated by the following equation:

(3) $$\begin{array}{c} \left(1\right)IM=\overset{\infty }{\underset{i-1}{\sum }}M^{i}=M^{2}{\left(I-M\right)}^{-1}\text{.} \end{array}$$

To calculate the total-influence matrix, the value of the total-influence matrix can be obtained from the value of the direct-influence matrix, and the value of the indirect-influence matrix can be calculated using the following equations:

(4) $$\begin{array}{c} \left(2\right)T=M+IM=\overset{\infty }{\underset{i=1}{\sum }}M^{i}\text{,} \end{array}$$

(5) $$\begin{array}{c} \left(3\right)T=\overset{\infty }{\underset{i=1}{\sum }}M^{i}={M\left(I-M\right)}^{-1}\text{.} \end{array}$$

Subsequently, the structural relationship between the factors is analyzed.

The sum vector of the row value is *d*_*i*_, and the sum vector of the column value is *r*_*i*_. Then, if we let *i* = *j*, the sum vector of the row value plus the column value will be (*d*_*i*_+*r*_*i*_), which represents the center degree. If the sum of the row value plus the column value (*d*_*i*_+*r*_*i*_) is high; thus, the relationship among dimensions or criteria will be powerful. The sum of the row value minus the column value is (*d*_*i*_ − *r*_*i*_), which indicates the extent of the reason. If *d*_*i*_ − *r*_*i*_ > 0, then the degree of influence on others is stronger than the degree of being influenced; otherwise, *d*_*i*_ − *r*_*i*_ < 0. Finally, the center degree (*d*_*i*_+*r*_*i*_) is taken as the *X* axis and the reason degree (*d*_*i*_ − *r*_*i*_) is taken as the *Y* axis.

In this study, the structure influence relation diagram was drawn. Next, the relation diagram was divided into four quadrants by the average of the center and reason degrees. The distributions of the indices were observed on the influence network diagram, and the causality and core degree of the index were analyzed.

### 3.4. FIA Model

Martilla et al. originally proposed the importance-performances (IPA) model to verify the importance and performance of factors being investigated, thereby dividing the two axes into four quadrants and indices [32]. Based on this model, decision-makers can sort through and improve the relevant attributes of their products or services. The IPA model does not waste resources on inappropriate and informal strategies and has long been considered a simple and effective technique. The present study extended its analysis of the FI and II. As shown in Figure 2, four frequency quadrants were constructed with frequency indicators based on the weighted survey provided by the respondents, and the impact indicates decision-makers to make strategic decisions. This study proposed four service improvement strategies for analyzing the four frequency and impact indicators.

  Priority: The first quadrant illustrates a high level of frequency and impact (H, H). This quadrant demonstrates that a factor has a high frequency and a high impact. Thus, medical device companies can prioritize solving this factor to strengthen their design development. In this research, we named this quadrant “Priority.”
  Investing resource: The second quadrant illustrates a low level of frequency and a high level of impact (L, H). The quadrant demonstrates that a factor has a high impact but does not reflect frequency. Therefore, medical device companies should invest resources in response to this factor. In this research, we named this quadrant “Investing resource.”
  Standstill: The third quadrant illustrates a low level of frequency and a low level of impact (L, L). This quadrant shows that factors situated in it have a low frequency and a low impact; thus, medical device companies can maintain their current status. In this research, we named this quadrant “Standstill.”
  Suspension: The fourth quadrant illustrates a high level of frequency and a low level of impact (H, L). This quadrant shows that the impact is not large, but the frequency is high. Medical device companies can suspend processing first. In this research, we named this quadrant “Suspension.”

### 3.5. NRM Analysis

The purpose of the DEMATEL method is to form a network diagram (i.e., an NRM). In addition, the method is mainly used to determine if factors interact or are independent, and the NRM is the final step in the DEMATEL method. The relationship between the degree and level of interaction of factors can be described by an easy-to-understand structure and a precise simplification of interdependence [33]. The NRM differs from the FIA model in the sense that it assigns and ranks factors based on specific characteristics. The NRM reveals the interrelationships among factors and evidence that provides additional important factors. A structural matrix and causal map can be used to show causality and impact, and the factors in a complex system can promote decision-making [34, 35].

## 4. Data Analysis and Results

### 4.1. Content Analysis

Based on the literature review, case studies and interviews with experts, the process of medical device development is divided into user action (UA), technical capability (TC), use environment (UE), and organizational characteristics (OC). To answer our research question (what are the challenges in the development of medical devices?), we interviewed experts with experience in medical device development in Taiwan. These experts come from a variety of medical device-related organizational backgrounds, including audit organizations, consulting firms, government agencies, and medical device companies. For this study, a minimum of six years of experience in the development or evaluation of multiple medical devices is required for someone to be called an expert. The respondents were interviewed face-to-face with informed consent in order to understand the key factors in the development of current medical devices. An overview of the stakeholders is provided in Table 1. Three experienced coders are responsible for the verbatim coding of the interviews for content analysis. The UA, TC, UE, and OC profiles and 16 key factors were extracted from the interviews and cited in the literature or the expert interviews. In addition, these key factors were clearly defined and analyzed for reliability (Table 2). Three coders performed the coding. Coders have experience in medical device innovation and underwent several rounds of practice coding with subsamples. Coders calculate the number of factors that each coder overlapped and then calculate mutual agreement and reliability. Disagreements were resolved after discussions and reassessments of the case to eventually arrive at a consensus.  Table 3 shows that the average mutual agreement between the coders is 0.844, which is high. In addition, the reliability test presents that the reliability of the three coders interviewed is 0.942, and the values greater than 0.8 represent the high reliability of content analysis [36].

### 4.2. FIA-NRM Model

The purpose of FIA is to conduct placement positioning based on the dimensions and the factors FI and II such that the medical device developers can have an adequate command of the frequency and impact of each dimension or factor. To build the FIA models, the average values of the weights (from 0 to 10 points) provided by the respondents to the criteria are calculated and standardized using standard deviation. Each criterion has one frequency value and one impact value, which helps determine its position in the FIA model. NRMs are developed using the DEMETAL method to present the causal relationship and the degree of impact between the dimensions and barriers in a complex system, which can facilitate the decision-making process. Criteria with high (*d* + *r*) values have strong relationships with other criteria, whereas those with low (*d* + *r*) values have weak relationships with other criteria. Furthermore, criteria with a positive (*d* − *r*) can influence other criteria, whereas those with a negative (*d* − *r*) have a high chance of being influenced by others.

Based on the reliability and validity analysis, the Cronbach's alpha of the primary dimension is 0.959, the Cronbach's alpha of UA is 0.886, the Cronbach's alpha of TC is 0.872, the Cronbach's alpha of UE is 0.906, and the Cronbach's alpha of OC is 0.871. The results show that the research questionnaire demonstrates high reliability (Table 4).

#### 4.2.1. Primary Dimensions

Primary dimensions, including UA, TC, UE, and OC, were analyzed in the FIA model, which is characterized by levels of impact and frequency.  Figure 3 and Table 5 reveal that TC has a high impact and high frequency; thus, priority should be given immediately. OC and UA have a high impact but low frequency; thus, considerable resources and efforts should be invested to abolish factors. Finally, UE has a low impact and low frequency; thus, developers can maintain standstill action. Therefore, developers should prioritize the following order of the dimensions: TC ⟶ OC ⟶ UA ⟶ UE. As for the NRM model, Figure 4 and Table 5 indicate that UA demonstrates the highest (*d* + *r*) value and the strongest connection with the other dimensions. Furthermore, UA has a positive (*d* − *r*) value, and thus has a remarkable impact on the other dimensions. For further observations on the causal relationships between the primary dimensions, Table 6 provides data on their net influence. Table 6 points out that OC influences all the other dimensions, TC influences UA and UE, and UE influences UA.

Figure 4 shows that four improvement pathways exist via NRM analysis, that is, OC ⟶ UA, OC ⟶ TC ⟶ UA, OC ⟶ UE ⟶ UA, and OC ⟶ TC ⟶ UE ⟶ UA. Tables 5 and 6 demonstrate that the ranking of the FI is TC > UE > OC > UA, and the ranking of the II is TC > UA = OC > UE. To find a possible pathway, a dimension with a high rank is used to affect a dimension with a low rank. For example, in FI, the second pathway, that is, TC (ranked 1) can improve UA (ranked 4), and this pathway will be accepted. The remaining pathways also follow this logic. Four solvable pathways exist in the FI, and four solvable paths likewise exist in the II. Next, we find four overlapping solvable pathways, as shown in Table 7. Table 7 summarizes the improvement paths and recommended pathways that medical device developers can follow to solve the main dimensions of medical device development.

1. Developers should efficiently take investing resources to improve OC to determine UA.
2. Developers should efficiently take investing resources to improve OC, then take priority action to ameliorate TC to determine UA.
3. Developers should efficiently take investing resources to improve OC, then take standstill action to define UE to determine UA.
4. Developers should efficiently take investing resources to improve OC, take priority action to ameliorate TC, then take standstill action to define UE to determine UA.

#### 4.2.2. User Action Dimensions

Four categories comprised of UA, namely, the user needs considerations (UA1), training course (UA2), empirical cognitive ability (UA3), and physical and mental health (UA4).  Table 8 and the FIA model in Figure 5 indicate that UA1 and UA2 have a high frequency and high impact. Hence, developers should prioritize solving these two categories immediately. As UA3 has a high impact but low frequency, developers can assess the investment of resources. Finally, the low levels of impact and frequency of UA4 suggest standstill action. Developers are recommended to prioritize the following order of the factors: UA1 ⟶ UA2 ⟶ UA3 ⟶ UA4.

As for the NRM model, Figure 6 reveals that UA4 influences all the other UA categories, UA1 influences UA3 and UA2, and UA3 influences UA2.

Figure 6 and Table 8 show that the ranking of the FI is UA1 > UA2 > UA3 > UA4, and the ranking of the II is UA1 > UA3 > UA2 > UA4. Two solvable pathways are observed in the FI, and three solvable paths are seen in the II. Next, we find two overlapping recommended pathways: UA4 ⟶ UA1 ⟶ UA2 and UA4 ⟶ UA1 ⟶ UA3 ⟶ UA2.

#### 4.2.3. Technical Capability Dimensions

There were four categories that comprised TC, namely, user interface design (TC1), competitive products (TC2), calibratable maintenance (TC3), and label warning (TC4).  Table 9 and the FIA model in Figure 7 indicate that TC1 and TC4 have a high frequency and high impact. Hence, developers should prioritize solving these two categories immediately. As TC2 has a high impact but low frequency, developers can assess the investment of resources. Finally, the low impact and high frequency of TC3 suggest the suspension of action. Developers are recommended to prioritize the following order of the factors: TC1 ⟶ TC4 ⟶ TC2 ⟶ TC3. As for the NRM model, Figure 8 reveals that TC1 influences all the other TC categories, TC2 influences TC3 and TC4, and TC3 influences TC4.

Figure 8 and Table 9 demonstrate that the ranking of the FI is TC4 > TC3 > TC1 > TC2 and the ranking of the II is TC1 > TC2 > TC4 > TC3. Two solvable pathways exist in the FI and four solvable paths exist in the II. We find two overlapping recommended pathways: TC1 ⟶ TC2 ⟶ TC4 and TC1 ⟶ TC2 ⟶ TC3 ⟶ TC4.

#### 4.2.4. Use Environment Dimensions

UE is comprised of four categories, namely, intended location (UE1), public safety protection (UE2), hygiene requirements (UE3), and device usage time (UE4).  Table 10 and the FIA model in Figure 9 indicate that UE1 and UE4 have a low impact but high frequency, thereby suggesting the suspension of action. The low levels of impact and frequency of UE2 and UE4 suggest that standstill action should be taken. Developers are recommended to prioritize the following order of the factors: UE1 ⟶ UE4 ⟶ UE2 ⟶ UE3. As for the NRM model, Figure 10 reveals that UE1 influences all the other usage barriers, UE4 influences UE2 and UE3, and UE2 influences UE3.

Figure 10 and Table 10 demonstrate that the ranking of the FI is UE4 > UE1 > UE2 > UE3, and the ranking of the II is UE3 > UE1 > UE2 > UE4. Three solvable pathways are seen in the FI, and three solvable paths exist in the II. We found three overlapping recommended pathways: UE1 ⟶ UE4 ⟶ UE3, UE1 ⟶ UE2 ⟶ UE3, and UE1 ⟶ UE4 ⟶ UE2 ⟶ UE3.

#### 4.2.5. Organizational Characteristic Dimensions

OC had four categories, namely, management culture (OC1), team communication (OC2), resource allocation (OC3), and regulatory standards (OC4).  Table 11 and the FIA model in Figure 11 indicate that OC4 and OC2 have a high frequency and high impact. Hence, developers should prioritize solving these two categories immediately. The low levels of impact and frequency of OC1 and OC3 suggest that standstill action should be taken. Developers are recommended to prioritize the following order of the factors: OC4 ⟶ OC2 ⟶ OC3 ⟶ OC1. As for the NRM model, Figure 12 provides data on their net influence.  Table 11 presents that OC1 influences all the other OC1 categories, OC2 influences OC4 and OC3, and OC4 influences OC3.

Figure 12 and Table 11 demonstrates that the ranking of the FI is OC4 > OC2 > OC3 > OC1, and the ranking of the II is OC4 > OC2 > OC3 > OC1. Three solvable pathways exist in FI, and three solvable paths are observed in II. We identified three overlapping recommended pathways: OC1 ⟶ OC2 ⟶ OC3, OC1 ⟶ OC4 ⟶ OC3, and OC1 ⟶ OC2 ⟶ OC4 ⟶ OC3.

Recommended pathways based on the results of each of the above factors and tables and planning for the overall improvement path are shown in Table 12. The recommended improvement pathway order is OC ⟶ TC ⟶ UE ⟶ UA. Medical device developers should examine and analyze each factor. A range of informal and formal organizational processes can influence user considerations, user interfaces, and UE in the development of medical devices. Moreover, adopting a formal decision-making process can help medical device developers develop an integrated and reflective approach to improve business decisions and quality end products.

## 5. Discussion

This study clarifies the key factors of the medical device development process from the user and stakeholder perspectives. In addition, this study analyzes the frequency and impact of these critical factors on the medical device development process and suggests strategies for improvement.

### 5.1. Theoretical Implications

This study fills the research gap in key factors that affect the development of medical devices and improvement paths. The FIA results indicate that medical device development stakeholders consider OC as the focus of medical equipment development. Consistent with the views of medical device regulatory authorities, the results demonstrate the importance of the safety and effectiveness of medical devices, including well-designed human-computer interface interaction based on user needs and conditions, and clearly defined product use information that includes mentioning warnings (based on product functions). Medical devices must comply with regulations before they can be marketed, and a recall mechanism should be in place in case of efficacy and safety concerns after marketing. Inappropriate medical devices will be deregulated or banned from the market because they often cause harm to end-users [41].

Although medical device development stakeholders consider UA and OC as infrequent problems, the two dimensions nonetheless exerts a large impact on medical devices. Numerous studies have noted that shortcomings still exist in the design of medical devices in terms of usability from users' perspectives, such as balancing conflicting user needs and ethical privacy [4, 48]. Medical device developers should identify priority input considerations as early as possible to satisfy user needs and provide education, training, and safety guidelines from the users' perspective [49]. This recommendation is also consistent with stakeholders' views that UA considerations should focus on satisfying user needs and improving training courses, whereas the assessment of user background and individual physical and mental status is difficult and not a priority in the product development process. OC aspects, including regulatory standards and team communication, from medical device design to market entry, are also important in the development and profit of medical devices. Team communication within organization is critical [50]. Moreover, owing to the particularity of medical devices, regulatory standards have become a key consideration in the marketing of medical devices. Medical device enterprises should familiarize themselves with national regulations as well as the economic status and social backgrounds of their targeted market as early as possible [9] and develop their product listing process and market plans. Finally, medical device company stakeholders believe that UE is not a priority in the product development process. This finding may be due to the strict regulatory mechanisms of medical devices for product safety specifications; thus, parameter settings and range have been applied to most environmental factors.

### 5.2. Practical Implications

Medical devices make resource input in its development process far higher than that of general products. Compared with large enterprises, SMEs are disadvantaged in terms of risk control, manufacturing, and operation performance owing to insufficient resources [51]. This finding has made it necessary for numerous SMEs that manufacture medical devices to evaluate resource planning strategies and develop appropriate paths for product development and healthcare benefits in the context of limited resources [52, 53]. Based on the views of stakeholders on the development of medical devices, this study proposes development order and path suggestions in the development of medical devices (Figure 13). The results of this study suggest that medical device development strategies should improve management culture and team communication within the organization and allocate development resources after confirming medical device regulatory standards. After confirming the feasibility of development, medical device developers need to consider the user interface design in terms of technical capability, establish calibration and maintenance standards, and label warnings on their products. Next, medical device developers need to consider the impact of the surrounding environment on the device, including the location, time of use, protective facilities, and hygiene requirements. Finally, even though medical regulations have established the safety and usability of medical devices, medical device developers must still take into consideration the unique circumstances of possible users.

The development of medical devices is usually for start-up teams or SMEs. The establishment of a climate of intense collaboration and communication between different areas of the organization not only facilitates motivated new projects and rapid decision-making, but also focuses on user needs from concept to disposal of the product lifecycle and integrates the development process, which is an important basis for the development of medical devices [54]. Due to the complexity of the multisite, multiperson, and multidevice context of many medical interactions, the ensuing user behaviour can have a range of implications for the effectiveness of medical procedures. Developers need to design user interfaces based on technical features, in particular to understand the ergonomic impact of products and clinician/nursing staff interactions with patients based on information from competing products, and to establish product maintenance and warning standards [55]. The clinical environment usually involves at least two participants in the interaction (clinician and patient) and there are often many complex environmental factors that affect the overall procedure or task, such as the conditions of use of the device (e.g., portability, manoeuvrability, conflict of existing equipment and use of power outlets), the physical environment (e.g., the impact of bedrail design on patient behaviour), and the size of the space available may all limit the usability of the medical device. Developers should therefore also consider the impact of environmental factors on the use of the device when assessing the overall outcome of the device design. Finally, although all of the above factors are met, a medical device is considered marketable. However, the findings of this study suggest that it would be helpful if the development team could take into account the user's condition, including physical and mental health, needs, and training. For example, the packaging of disposable devices may affect the time and efficiency pressures on medical staff, while the sensitive clinical nature of ultrasound is crucial to the physical and psychological comfort of patients. In addition, in the case of long-term health outcomes, other factors of the patient (age, clinical condition, and medication effects) may be no less influential than the design of the device [55]. This inside-out process of influence is a key in the development of numerous enterprises [5, 56] and covers various fields. Thus, in the present study, the proposed development paths of medical devices from the perspective of stakeholders can be seen as logical and valuable.

## 6. Conclusion

This study uses content analysis and FIA-NRM to discuss stakeholders' views on key factors in medical device development. This study summarizes important factors in the development of medical devices and the views of various stakeholders. This research suggests that the development of medical equipment should start with OC and strengthen TC. Next, according to the evaluation indicators of this study, medical device developers can consider UA and UE strategies and improve functional design, product safety, and clinical application planning with optimal resource allocation. In the future, this study will be able to incorporate input from other stakeholders, including healthcare providers, venture capitalists, and government agencies. It will also be able to conduct case studies on different medical device categories. In the long run, the medical device development strategies developed in this study can benefit the medical industry, health care policy, and national development.

## Figures and Tables

**Figure 1:** Research framework flowchart.

**Figure 2:** FIA model.

**Figure 3:** Main dimensions' FIA model of medical device development.

**Figure 4:** Main dimensions' NRM model of medical device development.

**Figure 5:** FIA model for UA.

**Figure 6:** NRM model for UA.

**Figure 7:** FIA model for TC.

**Figure 8:** NRM model for TC.

**Figure 9:** FIA model for UE.

**Figure 10:** NRM model for UE.

**Figure 11:** FIA model for OC.

**Figure 12:** NRM model for OC.

**Figure 13:** Medical device development strategy.

**Table 1:** The interviewee's background information.

	Organization background	Position	Experience with medical device (years)	Interview time (min)
Expert 1	Auditing organizations	Manager	12	45
Expert 2	Auditing organizations	Manager	15	60
Expert 3	Consultant company	CEO	8	30
Expert 4	Government agency	Manager	6	45
Expert 5	Government agency	Manager	8	45
Expert 6	Medical device company	Product manager	6	55

**Table 2:** Assessment structure of medical device development.

Dimension	Factor	Description	Literature	Interview
User action (UA)	User needs considerations	Plan product designs that meet target users' needs with the intended use and service capabilities	A	●
	Training course	Education and training courses for users to avoid errors and failures in use	B	●
	Empirical cognitive ability	Users need to have basic knowledge and experience to avoid misuse of the product	C	●
	Physical and mental health	Product function design is based on the user's physical health and mental state	D	

Technical capability (TC)	User interface design	Planning the human-machine interface design to meet safety regulations and user requirements	E	●
	Competitive products	The design is based on the published information and “recall” reports of the comparison products	F	●
	Calibratable maintenance	Functional testing, calibration maintenance, and troubleshooting specifications for products	GH	●
	Label warning	According to the product's attribute type and service function, design a clear label warning	IJ	●

Use environment (UE)	Intended location	Product placement is evaluated based on the intended environment and conditions of use	K	●
	Public safety protection	Planning protective measures according to formulate safety operation rules to prevent accidents	L	●
	Hygiene requirements	Develop clean and hygienic requirement standards for the use of the environment	MN	
	Device usage time	Make reasonable operating procedures based on the length of usage time for the product	OP	●

Organizational characteristic (OC)	Management culture	Different organizational management models and cultures influence product design	Q	●
	Team communication	Communication within and outside of the organization affects the development of products	R	●
	Resource allocation	Planning for the allocation of resources to support all phases of product development	ST	●
	Regulatory assessment	Setting product design strategies to meet regulatory requirements of medical device quality control	U	●

Note: A: [14], B: [15], C: [16], D: [37], E: [38], F: [39], G: [8], H: [40], I: [41], J: [42], K: [17], L: [18], M: [43], N: [44], O: [19], P: [20], Q: [45], R: [46], S: [47], T: [21], U: [9].

**Table 3:** Reliability and mutual agreement between coders.

	Coder 1	Coder 2
Coder 3	0.828	0.839
Coder 2	0.867	—
Average mutual agreement: **0.844**		Reliability: **0.942**

0.844 indicates high agreement between coders for content analysis. 0.942 is greater than 0.8 indicating high reliability of content analysis.

**Table 4:** Reliability and validity analysis.

Dimension	Alpha	Test result
Main dimensions	0.959	Highly creditable
UA	0.886	Highly creditable
TC	0.872	Highly creditable
UE	0.906	Highly creditable
OC	0.871	Highly creditable

*Note.* Cronbach's *α* values show that *α* < 0.35 is lowly creditable, 0.35 < *α* < 0.7 is moderately creditable, and *α* > 0.7 is highly creditable.

**Table 5:** Statistical analysis and strategy for main dimensions.

Dimensions	FIA			NRM			Strategy
	FI	II	(FI, II)	*d* + *r*	*d* − *r*	(*d* + *r*, *d* − *r*)	
UA	−0.801	0.215	(L, H)	27.059	−0.193	(+, +)	Investing resource
TC	1.450	0.971	(H, H)	26.837	0.003	(+, −)	Priority
UE	−0.172	−1.402	(L, L)	24.687	−0.035	(+, −)	Standstill
OC	−0.477	0.215	(L, H)	23.931	0.226	(+, +)	Investing resource

*Note.* L stands for “low” and H stands for “high.”

**Table 6:** Net influence matrix for primary dimensions.

Net influence matrix	UA	TC	UE	OC
UA	—			
TC	0.055	—		
UE	0.038	−0.017	—	
OC	0.101	0.068	0.057	—

**Table 7:** Recommended pathways for solving main dimensions.

	FI	II
Rank	TC [1] > UE [2] > OC [3] > UA [4]	TC [1] > UA [2] = OC [2] > UE [3]

Improvement pathways	(1) OC [3] ⟶ UA [4]	(1) OC [2] ⟶ UA [2]
	(2) OC [3] ⟶ TC [1] ⟶ UA [4]	(2) OC [2] ⟶ TC [1] ⟶ UA [2]
	(3) OC [3] ⟶ UE [2] ⟶ UA [4]	(3) OC [2] ⟶ UE [3] ⟶ UA [2]
	(4) OC [3] ⟶ TC [1] ⟶ UE [2] ⟶ UA [4]	(4) OC [2] ⟶ TC [1] ⟶ UE [3] ⟶ UA [2]

Recommended pathways	(1) OC ⟶ UA	
	(2) OC ⟶ TC ⟶ UA	
	(3) OC ⟶ UE ⟶ UA	
	(4) OC ⟶ TC ⟶ UE ⟶ UA	

**Table 8:** Statistical analysis and strategy for UA.

Dimensions	FIA			NRM			Strategy
	FI	II	(FI, II)	*d* + *r*	*d* − *r*	(*d* + *r*, *d* − *r*)	
UA1	1.260	1.850	(H, H)	43.556	−0.165	(+, −)	Priority
UA2	0.026	0.123	(H, H)	43.083	−0.260	(+, −)	Priority
UA3	−0.420	0.203	(L, H)	43.412	−0.188	(+, −)	Investing resource
UA4	−2.306	−1.765	(L, L)	37.847	0.613	(+, +)	Standstill

**Table 9:** Statistical analysis and strategy for TC.

Dimensions	FIA			NRM			Strategy
	FI	II	(FI, II)	*d* + *r*	*d* − *r*	(*d* + *r*, *d* − *r*)	
TC1	0.609	1.007	(H, H)	28.818	0.539	(+, +)	Priority
TC2	−0.180	0.966	(L, H)	28.242	0.377	(+, +)	Investing resource
TC3	1.020	−0.520	(H, L)	27.343	−0.246	(+, −)	Suspension
TC4	1.157	0.404	(H, H)	26.955	−0.670	(+, −)	Priority

**Table 10:** Statistical analysis and strategy for UE.

Dimensions	FIA			NRM			Strategy
	FI	II	(FI, II)	*d* + *r*	*d* − *r*	(*d* + *r*, *d* − *r*)	
UE1	0.094	−0.600	(H, L)	44.307	0.207	(+, +)	Suspension
UE2	−0.180	−0.801	(L, L)	43.520	0.100	(+, +)	Standstill
UE3	−0.352	−0.359	(L, L)	43.014	−0.438	(+, −)	Standstill
UE4	0.129	−0.921	(H, L)	41.119	0.131	(+, +)	Suspension

**Table 11:** Statistical analysis and strategy for OC.

Dimensions	FIA			NRM			Strategy
	FI	II	(FI, II)	*d* + *r*	*d* − *r*	(*d* + *r*, *d* − *r*)	
OC1	−1.620	−1.042	(L, L)	26.210	0.513	(+, +)	Standstill
OC2	0.574	0.083	(H, H)	25.745	−0.009	(+, −)	Priority
OC3	−0.900	−0.319	(L, L)	25.547	−0.426	(+, −)	Standstill
OC4	1.089	1.689	(H, H)	23.040	−0.078	(+, −)	Priority

**Table 12:** Summary of improvement pathways.

Order	Dimension	Improvement pathways
1	OC	OC1 ⟶ OC2 ⟶ OC4 ⟶ OC3
2	TC	TC1 ⟶ TC2 ⟶ TC3 ⟶ TC4
3	UE	UE1 ⟶ UE4 ⟶ UE2 ⟶ UE3
4	UA	UA4 ⟶ UA1 ⟶ UA3 ⟶ UA2

## Data Availability

The data used in this article cannot be shared publicly due to privacy reasons of the participants of the study.
